# Livestock Drugs and Disease: The Fatal Combination behind Breeding Failure in Endangered Bearded Vultures

This article has been retracted.

**DOI:** 10.1371/journal.pone.0014163

**Published:** 2010-11-30

**Authors:** Guillermo Blanco, Jesús A. Lemus

**Affiliations:** Departamento de Ecología Evolutiva, Museo de Ciencias Naturales (CSIC), Madrid, Spain; University of Georgia, United States of America

## Abstract

There is increasing concern about the impact of veterinary drugs and livestock pathogens as factors damaging wildlife health, especially of threatened avian scavengers feeding upon medicated livestock carcasses. We conducted a comprehensive study of failed eggs and dead nestlings in bearded vultures (*Gypaetus barbatus*) to attempt to elucidate the proximate causes of breeding failure behind the recent decline in productivity in the Spanish Pyrenees. We found high concentrations of multiple veterinary drugs, primarily fluoroquinolones, in most failed eggs and nestlings, associated with multiple internal organ damage and livestock pathogens causing disease, especially septicaemia by swine pathogens and infectious bursal disease. The combined impact of drugs and disease as stochastic factors may result in potentially devastating effects exacerbating an already high risk of extinction and should be considered in current conservation programs for bearded vultures and other scavenger species, especially in regards to dangerous veterinary drugs and highly pathogenic poultry viruses.

## Introduction

Environmental pollutants are increasingly documented as a driver of wildlife endangerment due to their roles in organ damage, hormonal disruption and alteration of the immune system [1], [2]. Disease may also facilitate endangerment and extinction at global and local scales, especially when pathogens interact with other drivers such as pollutants [3]. There is increasing concern about the impact of veterinary drugs and livestock pathogens as factors damaging wildlife health [4]–[6], and even causing declines approaching extinction [7]. These threats may be especially detrimental to wildlife as they increasingly concur and interact as a consequence of the elimination of livestock residues containing veterinary pharmaceuticals and resistant pathogens due to growing intensive livestock operations worldwide [6], [8], [9]. In particular, the ingestion of antimicrobials, primarily fluoroquinolones, has been recently related to immunodepression-mediated acquisition of opportunistic pathogens and disease, as well as to organ damage in nestling vultures [6], [10], [11]. Fluoroquinolone residues have also been found in avian scavenger eggs and are associated with severe alterations in the development of embryo cartilage and bones that could preclude embryo movement and subsequently normal development, pre-hatch position and successful hatching [12]. Therefore, antimicrobials and other drugs may negatively affect embryo and nestling health with potentially devastating consequences on breeding success and conservation of vultures and other threatened avian scavengers.

The bearded vulture (*Gypaetus barbatus*) is one of the most endangered birds in Europe, with a main stronghold in the Pyrenees. Increasing declines in productivity (average number of fledglings raised per territorial pair) have recently been reported in the Spanish Pyrenees associated with habitat saturation processes [13], [14]. Given that bearded vultures may raise only one fledgling per breeding attempt, this productivity decline should be linked to increasing breeding failure when the proportion of territorial pairs that are breeding does not greatly vary with time [15]. The proximate mechanisms by which density can affect productivity have been investigated, including habitat heterogeneity, with progressively poorer territories being used, territory shrinkage and interference with breeders and floaters [13]. However, the proximate causes of breeding failure are poorly known despite the long-term interests in the conservation of this species [16]. To evaluate these causes, the examination of failed eggs and dead nestlings is imperative, including the study of the presence and impact of injury, developmental problems, poor nutritional condition, pollutants, organ damage, pathogens causing disease, etc. in order to determine the most likely cause of breeding failure.

Here, we conducted a comprehensive study of failed eggs and dead nestling bearded vultures collected during recent years in the Pyrenees. Both the productivity and survival rates of adults and young birds have reached the lowest values since the bovine spongiform encephalopathy (BSE) crisis [13], [14], [17]. This temporal decline could be related to illegal poisoning [17] and recent changes in the abundance, distribution and quality of carrion available to avian scavengers as a consequence of EU regulations derived from the BSE crisis [6], [18]–[20]. In particular, the BSE crisis caused the lack or scarcity of unstabled livestock available to scavengers and their subsequent increase in the consumption of carrion from stabled livestock, which is intensively medicated [21]. Therefore, we specifically focused on determining whether breeding failure in bearded vultures is related to the ingestion of veterinary drugs from stabled livestock carrion, as documented in other avian scavenger species [12]. We also assessed the potential effects of veterinary drugs on embryo damage and immunodepression increasing the probability of acquisition and proliferation of pathogens causing fatal disease [6], [10]–[12], [21]. Because veterinary drugs should be exclusively acquired from the ingestion of carrion from livestock medicated to combat disease, we predict that their presence should be associated with that of pathogens acquired from the same livestock, especially poultry pathogens more likely transmitted between avian species [22]. Alternatively, if the temporal decline in productivity was primarily associated with breeding failure due to the effects of habitat saturation processes [13], [17], we should expect egg and nestling mortality to be directly related to developmental and nutritional problems indicating progressively lower quality territories (e.g. embryo emaciation, nestling starvation) and interference by both conspecifics and heterospecifics (e.g. incubation failure, injury due to predation attempts or disturbance).

## Materials and Methods

Failed eggs (*n* = 5) and dead nestlings (*n* = 4) were collected from bearded vulture nests located in the Spanish Pyrenees between 2005 and 2008. The study of this material did not require of the approval of an ethics committee because it was collected after breeding failure (egg or nestling death) was confirmed in the field. Three of the specimens (two nestlings and one egg) were collected in 2005, 2007 and 2008 from a particular territory. Eggs and nestlings were collected after breeding failure and frozen. Necropsies were performed on all specimens according to standard protocols [12]. The age of embryos and nestlings were estimated according to size and development. Samples of liver, kidney, spleen, large and small intestines, lungs, brain, lymphoid organs (thymus, bursa of Fabricius, Peyer's patches) and knee joints were fixed in 10% buffered formalin, sectioned at 4 µm and stained for histopathological analysis [10], [12].

Liver (dead nestlings and failed embryos) and yolk (failed embryos) were used for the determination of the presence of veterinary drugs, including fluoroquinolones (enrofloxacin and ciprofloxacin), other antimicrobials (amoxicillin and oxytetracycline), non-steroideal anti-inflamatories (NSAIDs) such as diclofenac, flunixin meglumine, ketoprofen, ibuprofen, meloxicam, sodium salicylate, acetaminophen, and antiparasitics (metronidazole, diclazuril, fenbendazole, ivermectin) as described previously [12]. The limits of quantification, percentage recoveries, and inter- and intra-assay reproducibility were adequate [10], [12].

Other contaminants potentially affecting eggs and embryos were determined in liver, including heavy metals (Cd, Zn, Pb and Hg), following Blanco et al. [23], dithiocarbamate thiram, disulfuram, polybrominated diphenyl ethers, organochlorines and brominated flame retardants, following Lemus et al. [12] and carbamate and organophosphate pesticides (carbofuran, aldicarb and fenthion) following Elliot et al. [24]. We measured brain cholinesterase activity to assess early exposure to anticholinesterase pesticides [25]. Potential contamination was assessed by comparison with levels from apparently normal wild birds of other species [26] in the absence of basal levels for bearded vultures.

Determination of bacterial and fungal pathogens were conducted by sampling oropharynx, lung, liver, kidney, spleen, and intestine with sterile swabs and cultured using standard microbiology protocols [10], [12], [27], [28]. *Salmonella* serotypes and phage types were determined in the Spanish Reference Laboratory (Laboratorio Central Veterinario, Algete, Madrid). For confirmation of the identification of the alpha hemolytic *Streptococcus pneumoniae* we used a specific identification test (Accuprobe, Salem, MA) based on the detection of specific ribosomal RNA sequences. Samples of lesions found in internal organs and tissues during necropsies were taken with sterile swabs and cultured using the same standard microbiology protocols. In addition, we determined the presence of selected avian pathogens, including bacterial, viral, fungal, and protozoan pathogens by means of PCR-based methods (see Table S1 for details). The presence of *Chlamyophila psittaci* and *Mycoplasma* sp. in blood was determined as described previously [29], [30]. The presence of poxvirus, the paramyxovirus causing Newcastle disease, the serotypes H5, H7 and H9 of avian influenza, falcon adenovirus, circovirus, herpesvirus, polyomavirus, reovirus and West Nile virus were determined following the PCR-based methods available in the literature [31]–[39]. We also searched for helminths and protozoans in the gastrointestinal tract by macroscopic and microscopic observations using standard protocols [40].

Specific immunocytochemical procedures were used for detection of mielodepressive virus, including the alphaherpesvirus causing Marek disease [41] in kidney and bursa of Fabricius, the gyrovirus causing infectious chicken anaemia [42] in thymus and bone marrow, the birnavirus causing infectious bursal disease (IBD, [43]) in bursa of Fabricius, and the coronavirus causing chicken infectious bronchitis in kidney [44]. In addition, we conducted a specific immunocytochemical procedure for West Nile virus antigen detection [45] in brain, spinal medulla, thymus and thyroid. All immunohistochemistry analyses were conducted at the Department of Veterinary Anatomy, Veterinary Faculty, Universidad Complutense de Madrid, Spain and at the Pathology Department of the Veterinary Faculty, University of Utrecht, The Netherlands. The presence of these viruses was also determined by PCR-based methods [43], [46]–[48].

## Results

All dead nestlings and three of five unhatched embryos showed two to six different veterinary drugs in liver (nestlings) and egg yolk (embryos). In addition, the two embryos with fluoroquinolones in the yolk also had them in the liver (Table 1). Fluoroquinolones were the most prevalent drugs and showed the highest concentrations (Table 1). Other drugs such as NSAIDs and antiparasitics were found in most nestlings at variable concentrations, but in no eggs (Table 1). Other toxic compounds were detected in lower prevalence and concentrations (see Table 1 for those more relevant values; all insecticides were found at concentrations <0.001 ppb), which was further supported by basal levels of brain cholinesterase (Table 1).

**Table 1:** Presence and concentration (between brackets) of veterinary drugs, tissue damage and pathogens found in failed embryo and nestling bearded vultures.

Sample (Age)	Tissue for toxicology	Veterinary drugs^1^	Other toxicants^2^	Brain cholinesterase^3^	Pathology		Pathogen determination^5^	
					Tissue Damage^4^	Immunohistochemistry^5^	Microbiology	PCR
Nestling (35d)	Liver	EN (0.14), CI (0.03), OX (0.17), FL (32.48), AS (62.7), IV (5.4)	nondetected	17.15	UD, LE, LI, FN, BH, PK, GN, GO, MI, WP, ID^p^, JD	nondetected	CA, EC, SA* (septicaemia)	CH, WN
Nestling* (10d)	Liver	EN (0.11), CI (0.06), AS (47.9)	nondetected	16.24	UD, LE, BH, PK, GN, GO, MI, WP, ID^b,t,p^, JD	IBD	CA, EC	IBD
Nestling* (7d))	Liver	EN (0.08), CI (0.07), AS (37.4)	Pb (18.9)	18.42	UD, LE, BH, FN, PK, GN, MI, WP, ID^b,t^, JD	IBD	CA, EC, PM	IBD, WN
Embryo* (prehatch)	Liver	nondetected	OR (0.21), Pb (48.1)	15.37	UD, PK,MI, ID^p^	nondetected	CA	nondetected
Nestling (7d)	Liver	EN (0.03), CI (0.04), AS (52.3)	OR (4.9)	15.21	UD, LE, PK, GN, MI, WP, ID^b^, JD	IBD	CA, EC	IBD, WN
Embryo (prehatch)	Liver	nondetected	OR (0.88)	17.22	Endocarditis, leptomeningitis, PK, MI	BR	SS, SP (septicaemia)	BR
Embryo (mid incub.)	Liver Egg yolk	EN (0.06), CI (0.03) EN (0.04), CI (0.02)	nondetected	16.58	BH, FN, PK, GN, MI, WP, ID^b,p^, JD	IBD	SA**	IBD
Embryo (mid incub.)	Liver Egg yolk	EN (0.08), CI (0.03) EN (0.04), CI (0.05)	Pb (21.3)	18.11	BH, FN, PK, GN, MI, WP, ID^b,t^, JD	IBD	SA**	IBD
Embryo (mid incub.)	Liver Egg yolk	EN (0.05), CI (0.07) EN (0.07), CI (0.04)	nondetected	16.22	BH, FN, PK, GN, MI, WP, ID^b,t^, JD	IBD	SA**	IBD

Table 1 (cont.)

*Samples from the same territory in different years.

1 Veterinary drugs. EN: enrofloxacin (µg/g), CI: ciprofloxacin (µg/g), OX: oxytetracyclin (µg/g), FL: flunixin meglumine (µg/g), AS: sodium salicylate (ng/g), IV: Ivermectin (µg/g).

2 Other toxicants. OR: organochlorines (ng/g), Pb: lead (ng/g).

3 µmol/min/g

4 Tissue Damage. UD: upper digestive tract swelling, LI: liver lymphocytic infiltration, FN: focal liver necrosis, LE: liver enlarged, BH: bile duct hyperplasia, PK: pinkish kidney, GN: glomerullonephritis, GO: glomerullonephrosis, MI: mononuclear kidney infiltrates, WP: white kidney precipitates, ID: immunological tissue damage (b =  damage in Bursa of Fabricius, t =  damage in thymus, p =  damage in Peyer's patches), JD: joint damage.

5 Pathogens. CA: *Candida albicans*, EC: *Escherichia coli* enterotoxigenic, PM: *Pasteurella multocida*, SA*: Salmonella* (*Salmonella enterica enteritidis* 4, 5, 12: i: 1, 2, LT DT 104,

**Salmonella enterica enterica serotype Brancaster 4, 12. z29. SS: *Streptococcus suis*, SP: *Streptococcus pneumoniae*, CH: *Chlamydophila psittaci*, IBD: infectious bursal disease virus, BR: chicken infectious bronchitis virus, WN: West Nile virus.

Dead embryos and nestlings showed a moderate to good nutritional state. Major histopathological lesions were primarily located in the kidney, including glomerulonephritis and/or glomerulonephrosis present in all individuals with fluoroquinolones, but not in those without drugs (Table 1). All individuals with fluoroquinolones also showed joint lesions, including arthritis and/or arthrosis of the long bone articulations, as well as massive osseous stroma of the spongeous bones.

The fungi *Candida albicans* was isolated from the oral cavity of five individuals. All individuals showed non-specific mixed-bacterial flora. Enterotoxigenic *Escherichia coli* and *Salmonella* spp. were isolated in four cases (Table 1). *Salmonella* typing determined the presence of *Salmonella enterica enteritidis* 4, 5, 12: i: 1, 2, LT DT 104 (one case) and *Salmonella enterica enterica* serotype Brancaster 4, 12. z29 (three cases, see Table 1). One individual showed infection by *Salmonella enterica enteritidis* (see above) and enterotoxigenic *Escherichia coli* O86 in all examined organs (septicaemia) except brain, which rejected the possibility of post-mortem contamination. *Pasteurella multocida* was isolated in a single individual that also showed enterotoxigenic *Escherichia coli* O86 (Table 1); all of these individuals contained fluoroquinolones. One of the failed embryos without veterinary drugs showed suppurative myocarditis, multiple microabscesses in head muscles, suppurative leptomeningitis, as well as lower jaw gangrenous inflammation with loss of the osseous stroma due to a mixed infection with *Streptococcus suis* and *Streptococcus pneumoniae* in brain, meninges and neck muscles; this embryo also showed infection by chicken infectious bronchitis (Table 1). Both immunocytochemistry for the detection of poultry viruses and PCR pathogen survey were positive to IBDV in six individuals with fluoroquinolones (Table 1). Immunocytochemical procedures failed to detect West Nile virus antigens in individuals in which PCR for this virus had been positive. Parasitology was negative for all helminths, helminth eggs and protozoans.

## Discussion

We found multiple veterinary drugs, primarily fluoroquinolones, in most failed eggs and dead nestling bearded vultures from the Pyrenees. They also showed multiple internal organ damage and pathogens potentially acquired from medicated livestock carrion, especially viruses often infecting poultry. Recorded drug concentrations were among the highest reported in avian scavengers [6], [10]–[12], [21]. NSAIDs and antiparasitics were found in lower prevalence than fluoroquinolones, but at higher concentrations than those found in other avian scavengers, especially for flunixin meglumine and sodium salicylate [6], [12], [21]. On the contrary, we found no sterile eggs, poor nutritional conditions or injury in any failed embryo or nestling. Other pollutants were found in low prevalence and concentrations posing low risk to embryo and nestling health.

Fluoroquinolones may cause generalized direct developmental damage precluding embryo hatching, physiological alterations due to their impact on liver and kidney and immunodepression reducing resistance to opportunistic pathogens [6], [10]–[12], [21]. These pathogens may be acquired at the same time that drugs used to treat diseased livestock are ingested, as indicated by their high prevalence in embryos and nestlings. Therefore, despite the relatively small sample size resulting from low abundance, endangerment and logistic difficulties in reaching nests in this species, the results provide evidence of a combined impact of veterinary drugs and livestock disease as the primary cause of breeding failure in the sampled individuals.

The presence of West Nile virus is not likely to be associated with nestling disease or mortality because the lack of lesions in target tissues and viral antigen particles in the immunohistochemistry study. Fatal septicaemia caused by *Streptococcus suis*, one of the most important swine pathogens worldwide [49], in combination with septicaemia from *Streptococcus pneumoniae* and infection by chicken infectious bronchitis virus were found in a single embryo. This concentration of livestock pathogens has not been reported before and, to our knowledge, this is the first report of the three pathogens causing disease in a wild bird. Other pathogens recorded in embryos and nestlings, including *Salmonella* serotypes and phages typical of livestock [50], and enterotoxigenic *Escherichia coli* O86 causing septicaemia, were potentially transmitted by consumption of carcasses of infected poultry and other livestock [22], [27], [28]. In addition, we found that the IBD virus infected most individuals alone or together with other pathogens also potentially acquired from livestock carrion. This virus causes a highly contagious immunosuppressive bursal disease in poultry [51] and may be transmitted to wildlife in contact with poultry waste or by ingestion of carcasses [22], [52]. Nestlings are especially susceptible to IBD because of the primary role of bursa of Fabricius in immune function development at this age. In fact, immunosuppression due to IBD was indicated by the inflammation, necrosis and loss of lymphocytes in the bursa of Fabricius together with the presence of viral antigens recorded by means of immunocytochemical procedures. The potential impact of highly pathogenic and contagious poultry viruses has been previously recognized as a threat to wildlife health due to the increasing contact of wildlife with livestock operations in general, and poultry farms and their residues in particular, in natural areas worldwide [52]–[55]. However, damage from IBD virus on the bursa of Fabricius represents, to our knowledge, the first evidence of clinical disease compatible with death caused by this poultry virus in wildlife. The presence of IBD has been not previously recorded in embryos of wild birds, probably because vertical transmission has been ruled out in poultry and, as consequence, it has probably not been evaluated in other species until now. This striking and concerning result could be related to the longer egg development and incubation periods of bearded vultures compared with poultry, and/or due to contrasting environmental conditions during incubation between bearded vultures and poultry. Thus, embryo infection with IBD may occurs via the female or during incubation as a consequence of egg contact between the egg and poultry remains in the nests of bearded vultures, which requires more research.

Despite their potential effects on population dynamics and conservation through a reduction of productivity and changes in mating behaviour [13], [14], habitat saturation processes were apparently not directly related to particular proximate causes of egg and nestling failure in this study or in these sampled individuals. As an alternative non-mutually exclusive explanation, we suggest that the recent decline in productivity could also be linked to the increasing ingestion of veterinary drugs and acquisition of pathogens from medicated stabled livestock carcasses due to decreasing availability of unstabled livestock carcasses - the traditional primary food of bearded vultures [16]- since the BSE crisis [21], accompanied by a possible increasing use of antibiotics in stabled livestock operations. In this sense, it is remarkable that bearded vultures primarily feed upon livestock bones, which are one of the major target tissues of fluoroquinolones in medicated animals [56], therefore, rendering this species especially sensitive to the consequences of an increase in the consumption of stabled intensively medicated livestock. The presence of veterinary drugs in eggs implies their previous presence at least in breeding females [12], but also probably in breeding males and non-breeders frequently using artificial feeding sites and livestock carcass dumps [17], where veterinary drugs may be ingested from medicated livestock carcasses [10], [21]. Therefore, further research is required to determine the impact of veterinary drugs and livestock disease on fitness of full-grown individuals, including the potentially subtle, sublethal or indirect effects of these factors on population dynamics.

The link between veterinary drugs and livestock disease should be further investigated in scavenger species, because both threats may concur in food and because the immunodepressive effects and other physiological alterations caused by drugs may facilitate the acquisition and proliferation of pathogens [6], [11], [21]. Given that both threats acting together may greatly contribute to breeding failure decreasing productivity, their potential as stochastic factors with potentially devastating effects increasing the risk of extinction should be not overlooked in current conservation programs of bearded vultures and other scavenger species, especially regarding dangerous veterinary drugs and highly pathogenic viruses frequently infecting poultry. In addition, restricted geographic distribution and low genetic variability [57] common to many threatened species may favour pathogen transmission and reduce the ability of a naïve immune system to fight against novel pathogens [3], [28], [58], making them especially vulnerable to the potential cross-species transmission of highly virulent virus strains able to cause important outbreaks, as reported in poultry [59]–[61].

The association of pollution and disease may further increase extinction risk if it interacts with the effects of habitat saturation processes [13], [14], [17]. These processes may facilitate conspecific contact and interactions also likely to increase intra- and inter-specific pathogen transmission rates in breeding and feeding areas, especially of highly contagious poultry diseases [22]. This could be further enhanced by the artificially high numbers of bearded vultures and other scavengers attracted to feeding points and carcass refuse dumps, both as a result of management and due to the scarcity of unstabled livestock carcasses since the BSE crisis [17], [21]. Whatever the potential contribution of underlying ultimate mechanisms reducing productivity, our findings highlight the need to determine the proximate causes of breeding failure and mortality in wildlife populations in order to understand the processes regulating demography from an ecological framework perspective.

## Supporting Information

Table S1 (0.05 MB DOC)
